# Haplotype diversity and phylogenetic characteristics for Guanzhong Han population from Northwest China via 38 Y‐STRs using Yfiler™ Platinum Amplification System

**DOI:** 10.1002/mgg3.1187

**Published:** 2020-03-12

**Authors:** Luyao Li, Lilan Yao, Xin He, Huilin Gong, Yuan Deng, Mei Luan, Guanglin He, Fuquan Jia, Pengyu Chen

**Affiliations:** ^1^ Department of Pathology the First Affiliated Hospital of Xi'an Jiaotong University Xi'an Shaanxi China; ^2^ Center of Forensic Expertise Affiliated hospital of Zunyi Medical University Zunyi Guizhou China; ^3^ Department of Mathematics Sichuan University Chengdu Sichuan China; ^4^ Department of Dermatology and Venerology the First Affiliated Hospital of Xi'an Jiaotong University Xi'an Shaanxi China; ^5^ Institute of Forensic medicine West China School of Basic Science and Forensic Medicine Sichuan University Chengdu Sichuan China; ^6^ Department of Forensic Medicine Inner Mongolia Medical University Hohhot Inner Mongolia Autonomous Region China

**Keywords:** forensic genetics, genetic diversity, Guanzhong Han population, Y‐chromosomal STR, Yfiler™ Platinum system

## Abstract

**Background:**

For better application in human forensic cases and population genetics research, it is imperative to investigate the genetic characteristics of Guanzhong Han population using enhanced Y‐chromosomal short tandem repeats (Y‐STR) detecting system with higher discriminating power than previous ones.

**Methods:**

In this study, 38 Y‐STRs were profiled in 430 unrelated Chinese Han male individuals from Guanzhong region of Shaanxi Province, Northwest China, using the Yfiler™ Platinum PCR Amplification Kit. Haplotype frequencies and forensic parameters were calculated. Comprehensive population comparisons with geographically/ethnically different populations in China and other worldwide countries were performed.

**Results:**

A total of 422 different haplotypes were observed with the overall haplotype diversity (HD), discriminatory power (DC) and haplotype match probability (HMP) were 0.9999, 0.9814, and 0.0024, respectively. Guanzhong Han showed genetically affinity with Han ethnicity from Shanxi and Henan provinces, while far distant from Tibetan populations.

**Conclusion:**

This study offered a unique insight into Guanzhong Han population, the 38 Y‐STRs included in the the Yfiler™ Platinum system are highly polymorphic and informative and can be used for forensic practice and human genetic research.

## Graphical abstract

Thirty‐eight Y‐STR haplotype data in the Chinese Shaanxi Han population of 430 unrelated males were first reported using the Yfiler™ Platinum PCR Amplification Kit. Our findings in the present study indicated that the 38 Y‐STR loci were informative in the Guanzhong Han population and can be used as a powerful tool in forensic practice and population genetic study. Shaanxi Han showed genetically affinity with Han ethnicity from neighboring Shanxi and Henan province, while far distant from Tibetans in China.

## 1 BACKGROUND

Guanzhong, a basin located in the central part of Shaanxi Province, eastern Northwest China, consists of Xi'an, Xianyang, Baoji, Weinan, Tongchuan and Yangling (Figure 1). As one of the cradles of the Chinese civilization with a long history of more than 7,000 years, Guanzhong region was once the center of ancient Chinese Yellow River culture (Yang et al., 2008) and incubated the famous city—Chang'an (today's Xi'an), which was the origin of the Silk Road of China and, together with Athens, Rome and Cairo, shared the four ancient capitals of civilization in the world. Nowadays, Guanzhong is not only a key crossing place, linking to the road system of North and South Shaanxi, but also an important channel of cultural intercommunion and goods trade. The total population was 23.8506 million by the end of 2015 and Han population ranked as the first largest group (99.5%). People living there have distinctive dialect named Qin language, which belongs to the Sino‐Tibetan language family.

**Figure 1:** The geographical and ethnologic distribution of the investigated Guanzhong Han population and 19 other reference populations in China

Short tandem repeat located on the human Y chromosome (Y‐STR) loci with paternal lineage and haploid genetic feature, play a unique role in solving special forensic cases: revealing male donor of mixed stain for sexual assault cases, inferring paternal lineage origin and biogeographically ancestral information, and so on (Kayser et al., 2004; Purps et al., 2014). Over the past 20 years, a series of commercial kits consisting of varying number of Y‐STR loci were manufactured for forensic use. The Yfiler™ Platinum PCR Amplification Kit (Thermo Fisher Scientific) is a newly developed commercially available Y‐STR multiple detecting system, which could simultaneously amplify up to 41 forensically related Y chromosomal markers, including 38 Y‐STRs plus 3 Y‐InDels, with a six‐dye typing system over a read region of 60–565 bp. Because the included 38 Y‐STRs covering all markers currently designed in commonly used commercial Y‐STR kits, the Yfiler™ Platinum PCR Amplification Kit could be compatible with these previous developed kits and thus the corresponding historically male's profiles stored in national DNA database. Aforementioned studies have revealed that detecting more genetic markers of Y‐STR loci could evidently increase the discrimination power of unrelated males (Chen et al., 2018; Purps et al., 2014). So far, a great amount of Y‐STR haplotype data from geographically/ethnically different populations in China and other worldwide countries were reported to the Y‐STR Haplotype Reference Database (YHRD, https://www.yhrd.org), aiming at forensic and population genetics application in a specific population (Nothnagel et al., 2017; Purps et al., 2014). However, haplotype and forensic parameters of Y‐STRs in Han population from Guanzhong region of Shaanxi Province, Northwest China remain poorly investigated.

Herein, a study focusing on Guanzhong Han population analysis of Y‐chromosomal genetic diversity for 38 STR loci was conducted by the Yfiler™ Platinum system. We determined the haplotype diversity and forensic parameters of the 38 STR loci (DYS576, DYS389I, DYS635, DYS389II, DYS627, DYS549, DYS645, DYS460, DYS458, DYS19, YGATAH4, DYS448, DYS391, DYS557, DYS593, DYS522, DYS456, DYS390, DYS438, DYS392, DYS518, DYS444, DYS596, DYS570, DYS437, DYS449, DYS643, DYS393, DYS439, DYS481, DYS533, DYS447, DYS385, DYF387S1, and DYS527) and 3 Y‐InDels (rs771783753, rs759551978, and rs199815934) of the studied population. Then, population phylogenetic relationships exploration with geographically/ethnically distinct Chinese and world populations was performed.

## 2 METHODS

### 2.1 Sample preparation

A total of 430 unrelated Han male individuals were recruited who live in Guanzhong region of Shaanxi Province, Northwest China for at least three generations. Genomic DNA from blood samples was isolated using the Blood DNA Miniprep System (Promega) and the DNA concentration was quantified with Nanodrop‐2000 (Thermo Fisher Scientific) according to the manufacturer's instructions. The study was reviewed and approved by the Ethics Committee of Affiliated Hospital of Zunyi Medical University. For population genetic structure exploration, two reference population data sets were retrieved from the YHRD database (https://yhrd.org/), one consists of 19 other Chinese populations belonging to 13 ethnicities widely distributed in China, the other comprises 14 comparative populations around the world.

### 2.2 PCR amplification and genotyping

Thirty‐eight Y‐STR loci plus 3 Y‐InDels were co‐amplified using the Yfiler™ Platinum PCR Amplification Kit in a GeneAmp PCR 9700 thermal cycler (Thermo Fisher Scientific) following the manufacturer's instructions. Amplified fragments were detected by capillary electrophoresis on the Applied Biosystems 3500 Genetic Analyzer (Thermo Fisher Scientific). The electrophoresis data were automatically analyzed by GeneMapper^®^ ID‐X software (Thermo Fisher Scientific). Negative control (H_2_O) and positive control (007) were genotyped in each batch of DNA amplification. We strictly followed the recommendations for the DNA commission of the International Society of Forensic Genetics (ISFG) in the present study (Gusmao et al., 2006).

### 2.3 Statistical analysis

Allele and haplotype frequencies were determined by direct counting. genetic diversity (GD), haplotype diversity (HD) and haplotype match probability (HMP) were calculated using the following formulas: GD = *n* (1 − Σpiai^2^)/(n − 1), HD = *n* (1 − Σpihi^2^)/(n − 1), HMP = Σpihi^2^, where n represents the number of tested samples, and pi_ai_/pi_hi_ means the relative frequency of the i^th^ genotypes/haplotypes, respectively (Nei, 1981). The discrimination capacity (DC) was computed using the method by Purps (Purps et al., 2014). Population genetic comparisons between examined population and relative populations were performed using the analysis of molecular variance (AMOVA) in the website of YHRD (https://yhrd.org/amova), The genetic distance (Rst) and corresponding p values based on the 27 overlapped Y‐STRs were calculated. Multidimensional scaling analysis (MDS) was also constructed by aforementioned online tool on the basis of the Rst values.

## 3 RESULTS AND DISCUSSION

In the set of results, the haplotype distribution and frequencies are presented in Table S1. A total of 422 different haplotypes were identified from the 430 Guanzhong Han males, among which 415 different haplotypes were unique (98.34%), 6 different haplotypes were observed twice (0.46%), and 1 haplotype were observed three times (0.23%). No null allele was observed. Microvariant alleles were screened at one single‐copy locus DYS6450 and one multicopy locus DYS527. For DYS645, allele 6.4 was shared by six individuals. For DYS527, two intermediate alleles 20.2, 22.2 were identified, one allelic combination (20.2, 20.2) was found in six individuals, and the other allelic combination (22.2, 26) existed only once. Additionally, one triplicated allele (21, 22, 23) was also detected twice at DYS527.

Allele frequencies and the GD values of the 38 Y‐STR loci in 430 Guanzhong Han males are listed in Table S2. DYS385 was considered to be the highest locus (GD = 0.9635), whereas DYS645 was the lowest (GD = 0.0814) in Guanzhong Han population. The overall HD, DC, and HMP were found to be 0.9999, 0.9814, and 0.0024, respectively. Further comparisons of forensic statistical parameters based on varying STR number of 9, 12, 17, 23, 27, 29, and 38 included in MHT, PPY, Y filer, PPY23, Y filer plus, 29 Y‐STR level, and Y filer™ Platinum for our population data were summarized in Table S3. The results revealed that the percentage of detected unique haplotypes had remarkably raised from 74.56% (MHT) to 98.34% (38 STRs), and the 38 Y‐STR loci showed the highest haplotype diversity value (HD = 0.9999) and superior discrimination power (DC = 0.9814), which means a maximized distinction of unrelated males can be achieved by 38 Y‐STRs among all above Y‐STR kits. Generally, as the high performance of this Y‐Chromosome analysis system, 38 Y‐STR loci were highly polymorphic and informative in Guanzhong Han population and could be served as an effective tool for forensic practice and population genetic studies.

To further describe population genetic relationships, Rst and MDS were conducted based on the raw data of 27 overlapped Y‐STR loci with the online tool at YHRD. We first carried out population comparison at the domestic level. According to their geographic positions and ethnic origins, 19 previously reported Chinese populations belonging to Han majority and 11 ethnic minorities from distinct provinces were chosen as reference populations (see Figure 1), including 2 Han groups from Henan (Bai et al., 2016; Huang et al., 2019; Lang et al., 2019; Liu et al., 2019; Wang et al., 2016) and Shanxi (Sun et al., 2019), 5 Tibetan groups from Qinghai (Cao et al., 2018), Sichuan (Song, Xie, et al., 2019) Gansu and Tibet (Chamdo, and Shigatse), 3 Hui groups from Ningxia, Gansu (Liu et al., 2019; Ou et al., 2015; Xie et al., 2019), and Xinjiang (Zhang et al., 2019), Guizhou Bouyei (Feng et al., 2019), Guizhou Gelao (Liu et al., 2019), Hunan Dong (Luo et al., 2019), Hunan Yao, Hubei Tujia, Yanbian Korean, Hainan Li (Fan et al., 2018; Song, Wang, et al., 2019), Hulun Buir Mongolian (Wang et al., 2019), and Xinjiang Uighur. The pairwise genetic distance (Rst) with corresponding p values was listed in Table S4. There were no significant differences between Guanzhong Han and Shanxi Han and Ningxia Hui (*p* = .05/190 = 0.000263 after Bonferroni correction). The minimal genetic distance was observed with Shanxi Han (*R*st = 0. 0038), followed by Henan Han (*R*st = 0. 0081), while the largest genetic distance was found with 3 Tibetan populations from Sichuan (*R*st = 0.2388), Qinghai (*R*st = 0.1551), and Chamdo of Tibet (*R*st = 0.1421). As shown in Figure 2, Guanzhong Han closely clustered with Shanxi Han and Henan Han, as well as three Hui groups from different provinces (Ningxia, Gansu and Xinjiang) in the second quadrant, prominently distinguishing them from other minority groups. Most minorities from Southwest and South China mainly distributed in the third quadrant, such as Hunan Dong and Yao, Guizhou Gelao, and Bouyei, Hainan Li. While the other minorities from Northwestern China, including five Tibetan and one Uighur, were scattered in the first quadrants. Consistent with the aforementioned Rst values, MDS results revealed that Shaanxi Han showed genetically affinity with Han ethnicity from neighboring Shanxi and Henan provinces, while far distant from Tibetans in China.

**Figure 2:** The MDS showing the genetic relationships between the investigated population and 19 reference populations in China. The Guanzhong Han was marked in red

Further comparison at the worldwide level was implemented based on our investigated population with 14 representative populations from different continents and regions. As Rst and corresponding p values calculated in Table S5, statistical significance (*p* = .05/105 = 0.0005 after Bonferroni correction) was obviously displayed between Guanzhong Han and all others. Rst values ranged from 0.0585 (Guanzhong Han and Singapore Malay) to 0.2501 (Guanzhong Han and Ireland Irish [Aliferi et al., 2018]). As displayed in Figure 3, geographically related populations were prone to assemble together, and thus several typical clusters could be observed. Guanzhong Han along with the other two East Asian populations (Japan and South Kroean) scattered in the fourth quadrant. The cluster comprising three Southeast Asian populations (Philippines, Singapore and Laos), the cluster consisting three populations from East Europe (Russian), Northern Europe (Denmark), and Central Europe (Germany), as well as the cluster containing two South Asian populations (Indian and Afghanistan), separately concentrated on the first quadrant, second quadrant, and the upper side region in the MDS plot. Australian Europeans (Henry, Dao, Scandrett, & Taylor, 2019) and American Europeans closely group with each other, and then together with Australian aborigine on the fourth quadrant, which may be related to the common European ancestry origin between Australian Europeans and American Europeans, and the genetic flow between the Australian indigenous populations and the European immigrations for centuries. Among all compared foreign populations, Shaanxi Han had a closer relationship to East Asian.

**Figure 3:** The MDS between Guanzhong Han population and 14 reference populations around the world. The Guanzhong Han was marked in red

For comparisons based on both nationwide and worldwide, obvious geographic and ethnic cluster features were demonstrated in this study via MDS. In spite of this, the diminutive genetic distances were observed between Shaanxi Han and Northwest Chinese Hui. As Northwest China's major groups once active in the ancient silk road, Hui mixed dwelling with the Han population due to commercial logistics and marriage since the Tang Dynasty, and thus the two populations had a close genetic relationship (Xie et al., 2018). The previous results also confirmed that they have smaller genetic divergences (Purps et al., 2014).

## 4 CONCLUSION

In conclusion, this is a report to characterize the overall population and forensic genetics of Guanzhong Han population in China using Y‐STRs patterns. Our report disclosed the haplotype and forensic parameters based on 38 Y‐STR loci. The data showed highly polymorphic and informative in Guanzhong Han population and could be regarded as a valuable tool in forensic application and population genetic study. As a typical group residing in northwest area of China, population comparisons showed genetic affinity with geographic adjacent Han populations and remarkable genetic differentiation with Tibetan populations. Moreover, we observed Guanzhong Han had the close genetic relationship to East Asian populations by the result of genetic structure reconstruction, which indicated that the worldwide population substructures generally adhered to geographical distribution. For a better and in‐depth understanding of genetic background of Han population from Guanzhong region of Shaanxi province, more molecular genetic markers might be added in the future.

## CONFLICT OF INTEREST

No potential conflict of interest was reported by the authors.

## AUTHOR CONTRIBUTIONS

PYC and LYL conceived the idea for the study. FQJ, HLG, YD, and ML performed or supervised laboratory work. XH and GLH analyzed the data. PYC, LYL, and LLY wrote and edited the manuscript.
